This article has been retracted.

# LncRNA AWPPH promotes the growth of triple-negative breast cancer by up-regulating frizzled homolog 7 (FZD7)

**DOI:** 10.1042/BSR20181223

**Published:** 2018-11-28

**Authors:** Kainan Wang, Xuelu Li, Chen Song, Man Li

**Affiliations:** 1 Department of Oncology, Dalian Medical University, Dalian City, Liaoning Province 116044, P.R. China; 2 Department of Breast oncology, The Second Hospital of Dalian Medical University, Dalian City, Liaoning Province 116027, P.R. China

**Keywords:** AWPPH, frizzled homolog 7, LncRNA, proliferation, Triple-negative breast cancer

## Abstract

**Background:** LncRNA AWPPH is a recently identified critical player in the development of several types of human malignancies, our study aimed to investigate the role of AWPPH in triple-negative breast cancer. **Methods:** In the present study, expression of AWPPH in tumor tissues and adjacent healthy tissues of patients with triple-negative breast cancer as well as in plasma of both patients and healthy people was detected by qRT-PCR. Application potentials of AWPPH in the diagnosis and prognosis of triple-negative breast cancer were evaluated by ROC curve analysis and survival curve analysis, respectively. AWPPH expression vectors and frizzled homolog 7 (FZD7) siRNAs were transfected into cells of human breast cancer cell lines. Expression of FZD7 was detected by Western blot, and cell proliferation was detected using CCK-8 kit. **Results:** We observed that AWPPH was significantly up-regulated in tumor tissues than in paired adjacent healthy tissues of patients. Plasma levels of AWPPH were higher in patients than in controls. AWPPH overexpression promoted cancer cell proliferation and up-regulated FZD7 expression. FZD7 siRNA silencing inhibited cancer cell proliferation but did not significantly affect AWPPH expression. Compared with cells with AWPPH overexpression alone, cells with both FZD7 siRNA silencing and AWPPH overexpression showed significantly reduced proliferation ability. **Conclusions:** We conclude that LncRNA AWPPH may promote the growth of triple-negative breast cancer by up-regulating FZD7.

## Introduction

As one of the most common types of malignancy among females in the world breast cancer is responsible for 20% of deaths in women [1]. More and more studies have revealed that breast cancer is a heterogeneous disease that can be classified into different pathological subtypes with prognostic significance [2]. Categorization of breast cancer is mainly based on the expression of estrogen receptor (ER) and progesterone receptor (PR) and human epidermal growth factor receptor 2 (HER2) [3]. As a subtype of breast cancer, triple-negative breast cancer is characterized by the lack of ER and PR and the absence of HER2 overexpression [4]. Due to the extreme aggressive nature, low response rate to chemotherapy and lack of effective targeted therapies, prognosis of triple-negative breast cancer is generally poor [5].

The classic Wnt pathway plays pivotal roles in the development of different types of malignancies [6]. Wnt signaling is transduced through LRP5/lipoprotein receptor-related protein 6 (LRP6) co-receptor and Frizzled (FZD) family receptors to initiate the β-catenin signaling transduction [7]. As a critical player in Wnt pathway, frizzled homolog 7 (FZD7) has been proved to have pivotal functions in the regulation of cell proliferation in triple negative breast cancer [8]. It is known that Wnt pathway in some cases achieve its signaling transduction through the interactions with lncRNAs [9], which is a subgroup of non-coding RNA and plays pivotal roles in cancer biology [10]. AWPPH is a newly identified oncogenic lncRNA in bladder cancer [11] and hepatocellular carcinoma [12]. In our study, we observed that AWPPH might promote tumor growth in triple negative breast cancer by up-regulating FZD7.

## Materials and methods

### Specimens

Tumor tissue and adjacent healthy tissue specimens of 68 patients with triple-negative breast cancer, and plasma specimens of both patients and 62 healthy controls were obtained from the specimen library of the Second Hospital of Dalian Medical University. The 68 patients were diagnosed through pathological examinations and treated in the Second Hospital of Dalian Medical University from January 2010 to January 2013. Inclusion criteria: (1) patients diagnosed with triple-negative breast cancer by pathological examinations; (2) patients who were diagnosed and treated for the first time; (3) patients completed the whole treatment procedure; (4) patients with complete treatment and follow-up data. Exclusion criteria: (1) patients with other malignancies and other types of breast cancer; (2) patients transferred to other hospitals during treatment; (3) patients died of other causes during follow-up. Age of 68 patients ranged from 22 to 61 years, with a mean age of 40.2 ± 6.1 years. Age of 62 healthy females ranged from 24 to 63 years, with a mean age of 41.7 ± 5.4 years. No significant differences in age, BMI and other clinical data were found between two groups. The present study has been approved by the ethics committee of the Second Hospital of Dalian Medical University. Written form informed consent was obtained from all participants and/or their families. All experiments on human materials were performed in accordance with the World Medical Association Declaration of Helsinki.

### Real-time quantitative PCR

Total RNA extraction was performed using Trizol reagent (Invitrogen, U.S.A.) in strict accordance with manufacturer’s instruction. RNA with satisfactory quality was subjected to reverse transcription to synthesize cDNA. Systems of PCR reaction were prepared using SYBR Green PCR Master Mix (Thermo Fisher Scientific). Following primers were used in PCR reactions: 5′-CTGGATGGTCGCTGCTTTTTA-3′ (forward) and 5′-AGGGGGATGAGTCGTGATTT-3′ (reverse) for human lncRNA AWPPH; 5′-TTCTCGGACGATGGCTACC-3′ (forward) and 5′-GAACCAAGTGAGAGACAGAATGACC-3′ (reverse) for FZD7; 5′-GACCTCTATGCCAACACAGT3′ (forward) and 5′-AGTACTTGCGCTCAGGAGGA3′ (reverse) for β-actin. ABI PRISM 7500 sequence detection system (Applied Biosystems, Rockford, IL, U.S.A.) was used to perform all PCR reactions. PCR reaction cycles were: 95°C for 50 s, followed by 40 cycles of 95°C for 12 s and 60°C for 35 s. AWPPH expression was normalized to β-actin endogenous control using 2^−ΔΔ*C*^_t_ method.

### Cell lines, cell culture and transfection

Human triple negative breast cancer cell lines MDA-MB-231 and BT-20 were from ATCC. Cells of two cell lines were cultured with ATCC-formulated Eagle’s Minimum Essential Medium (Catalog No. 30-2003) containing 10% final concentration fetal bovine serum. Human FZD7 siRNA (Catalog # AM16708) and Silencer® Negative Control #1 siRNA (Catalog # AM4611) were from Thermo Fisher Scientific. DNA fragments containing full-length AWPPH or FZD7 cDNA surrounded by two *EcoRI* cutting sites were amplified through PCR using cDNA derived from human cells. The fragments were inserted into *EcoRI* linearized pIRSE2-EGFP vector (Clontech, Palo Alto, CA, U.S.A.) to construct AWPPH expression vector. Transfection was performed using Lipofectamine 2000 reagent (11668-019, Invitrogen, Carlsbad, U.S.A.) to transfect 10 mM vectors (10 nM) or 50 nM siRNAs into 5 × 10^5^ cells. Transfection efficiency was checked by qRT-PCR before subsequent experiments.

### Cell proliferation assay

Cell proliferation was detected by CCK-8 assay using a kit provided by Dojindo Molecular Technologies. Cell suspension with a cell density of 4 × 10^3^ cells/ml was prepared using cells of two cell lines. Then 4 × 10^3^ cells in 0.1 ml cell suspension was used to fill each well of a 96-well plate. Cells were cultured at 37°C with 5% CO_2_, and 10 μl of CCK-8 was added into each well at 24, 48, 72 and 96 h later. Cells were cultured for another 4 h and a microplate reader was used to measure OD values at 450 nm.

### Western blot

RIPA solution (Thermo Fisher Scientific) was used for all protein extractions in strict accordance with manufacturer’s instructions. BCA method was used to measure protein concentration. SDS-PAGE gel (10%) electrophoresis was then performed with 20 µg of protein per lane. Gel transfer was performed and PVDF membranes (Bio-Rad, U.S.A.) were incubated with skimmed milk (5%) for 2 h at room temperature for blocking. Membranes were then incubated with primary antibodies of FZD7 (rabbit anti human, ab64636, 1:1200; Abcam) and GAPDH (rabbit anti human, ab9485, 1:1200, Abcam) overnight at 4°C. Anti-rabbit IgG-HRP secondary antibody (1:1000, MBS435036, MyBioSource) was used to incubate with membranes the next day at room temperature for 2.5 h. ECL (Sigma-Aldrich, U.S.A.) was dropped onto membranes to develop signals, and ImageJ software was used to normalize FZD7 expression to GAPDH endogenous control.

### Statistical analysis

Graphpad Prism 6 software was used in the present study. Expression and cell proliferation data were recorded as mean ± standard deviation. Student’s *t* test was used for comparisons between two groups and comparisons among multiple groups were performed by one-way analysis of variance followed by Tukey test. Correlation analysis between AWPPH expression and patients’ clinicopathological data was performed by Chi-square test. *P*<0.05 was considered to be statistically significant.

## Results

### Comparison of AWPPH expression in tumor tissues and adjacent healthy tissues of triple-negative breast cancer patients

Differential expression of an lncRNA in tumor tissues and paired normal tissues indicates the involvement of this lncRNA in diseases. In the present study, expression of AWPPH in tumor tissues and paired normal tissues of 68 patients with triple-negative breast cancer was detected. As shown Figure 1, significantly up-regulated AWPPH expression in tumor tissues than in paired normal tissues was found in 57 out of 68 patients, accounting for 83.5%. Therefore up-regulated expression of AWPPH is likely involved in the pathogenesis of triple-negative breast cancer.

**Figure 1:** Comparison of AWPPH expression in tumor tissues and adjacent healthy tissues of triple-negative breast cancer *P<0.05.

### Comparison of plasma levels of AWPPH between patients and healthy controls and the potentials in disease diagnosis

Changes in circulating substances in blood usually reflect certain pathological changes. In the present study, AWPPH was detected in plasma of both 68 patients and 64 healthy controls. As shown in Figure 2A, plasma levels of AWPPH were found to be significantly higher in patients than in healthy controls (*P*<0.05). Potentials of AWPPH in the diagnosis of triple-negative breast cancer were explored by ROC curve analysis. Results showed that the area under the curve was 0.8927, with standard error of 0.02637 and 95% confidence interval of 0.8510 to 0.9444 (*P*<0.0001).

**Figure 2:** Comparison of plasma levels of AWPPH between patients and healthy controls and the potentials in disease diagnosis This figure shows the comparison of plasma levels of AWPPH between patients and healthy controls (**A**) and the potentials in disease diagnosis explored by ROC curve analysis (**B**). *P<0.05.

### Correlations between plasma levels of AWPPH expression and patients’ clinicopathological data

The 68 patients were divided into high and low expression groups according to the median plasma level of AWPPH, and correlation analysis between plasma levels of AWPPH and patients’ clinicopathological data was performed by Chi-square test. As shown in Table 1, plasma levels of AWPPH were not significantly correlated with age, BMI, smoking habit as well as existing of tumor distant metastasis. In contrast, a significant correlation was found between plasma levels of AWPPH and tumor size, indicating the potential involvement of AWPPH in tumor growth. In addition, plasma levels of AWPPH were also significantly correlated with TNM stages.

**Table 1:** Correlations between plasma levels of AWPPH expression and patients’ clinicopathological data

Variables	Groups	Cases	High expression	Low expression	χ²	*P* value
Age	>40 (years)	38	17	21	0.95	0.33
	<40(years)	30	17	13		
BMI	>24	27	12	15	2.32	0.31
	18.5–24	26	16	10		
	<18.5	15	6	9		
Smoking	Yes	22	10	12	0.27	0.60
	No	46	24	22		
TNM stage	I	12	3	9	9.38	0.02
	II	16	5	11		
	III	14	8	6		
	IV	26	18	8		
Primary tumor diameter	>5 cm	19	14	5	6.98	0.03
	2–5 cm	30	16	14		
	<2 cm	19	5	14		
Tumor distant metastasis	Yes	26	12	14	0.25	0.62
	No	42	22	20		

### Potentials of AWPPH in the prognosis of triple-negative breast cancer

Data in Table 1 showed no significant correlations between plasma levels of AWPPH and distant metastasis, which is responsible for more than 90% cases of cancer-related deaths. Therefore, AWPPH is unlikely involved in tumor metastasis and survival data of all patients were analyzed together. Kaplan–Meier method was used to plot survival curves for high and low expression groups and survival curves were compared by log rank *t* test. Results showed that overall survival of patients in low AWPPH expression group was significantly better than that of patients in high expression group (Figure 3, *P*<0.05).

**Figure 3:** Comparison of survival curves of low and high AWPPH expression groups

### Interactions between AWPPH and FZD7 in cells of human triple negative breast cancer cell lines

Our data showed that AWPPH is probably involved in the growth of triple negative breast cancer. It has been reported that FZD7 plays critical roles in cell proliferation of this disease. Therefore, potential interactions between AWPPH on FZD7 were explored. As shown in Figure 4A, AWPPH overexpression significantly promoted the expression of FZD7 in cells of both MDA-MB-231and BT-20 cell lines (*P*<0.05). In contrast, FZD7 overexpression showed no significant effects on AWPPH expression.

**Figure 4:** Interactions between AWPPH and FZD7 in cells of human triple negative breast cancer cell lines This figure shows the effects of AWPPH overexpression on FZD7 expression (**A**) and the effects of FZD7 overexpression on AWPPH expression (**B**). *P<0.05.

### Effects of AWPPH overexpression and FZD7 siRNA silencing on cell proliferation

*In vitro* cell proliferation results showed that AWPPH overexpression significantly promoted, while FZD7 siRNA silencing significantly inhibited the proliferation of cells of MDA-MB-231and BT-20 cell lines (Figure 5, *P*<0.05). In addition, compared with cells only transfected with AWPPH expression vectors, cells transfected with both AWPPH expression vectors and FZD7 siRNAs showed significantly reduced cell proliferation rate (Figure 5, *P*<0.05).

**Figure 5:** Effects of AWPPH overexpression and FZD7 siRNA silencing on cell proliferation of triple-negative breast cancer cell lines MDA-MB-231 (A) and BT-20 (B). *P<0.05.

## Discussion

The most important finding in our study is that AWPPH as a recently identified oncogenic lncRNA in bladder cancer [11] and hepatocellular carcinoma [12] may also play an oncogenic role in triple-negative breast cancer by promoting tumor cell proliferation. In addition, we also proved that the action of AWPPH in triple-negative breast cancer is probably achieved through the up-regulation of FZD7, which is a key player in Wnt signaling pathway.

Differential expression of a certain gene in lesion tissues and paired adjacent healthy tissues is a strong evidence of the involvement of this gene in human diseases. AWPPH was first identified as an oncogenic lncRNA overexpressed in hepatocellular carcinoma [12]. After that, overexpression of AWPPH has also been observed in bladder cancer tissues and cell lines [11]. In the present study, overexpression of AWPPH in tumor tissues than in adjacent healthy tissues was observed in most patients with triple-negative breast cancer, indicating that AWPPH may also be an oncogenic lncRNA in this disease. The fact that not all patients with triple-negative breast cancer show overexpression of AWPPH in cancer tissues indicates this molecular subtype of breast cancer may be also pathologically heterogeneous.

Pathological diagnosis is the gold standard for the diagnosis of most malignancies, while the invasive nature of this technique in some cases limits its application [13]. Changes in certain substances in blood with the development of human disease enable the use of circulating biomarkers in the diagnosis of human disease [14]. In our study, AWPPH was detected in the plasma of all patients with triple-negative breast cancer, and higher plasma levels of AWPPH were found in patients than in healthy controls. Further, ROC curve analysis also proved that up-regulation of AWPPH in plasma effectively distinguished triple-negative breast cancer patients from healthy controls. Besides that, plasma levels of AWPPH were not significantly correlated with age, BMI and smoking habits, which are verified prognostic factors for triple-negative breast cancer [15–17]. Those data suggest that AWPPH may participate in triple-negative breast cancer in a way independent from those factors.

Poor prognosis as main factor distinguished triple-negative breast cancer from other subtypes [18]. Tumor distant metastasis is the main cause of deaths in patients with malignancies [19]. In the present study, no significant correlations were found between plasma levels of AWPPH and the existing of distant tumor metastasis, while comparison of survival curves showed that up-regulated AWPPH expression is related to short survival time. Therefore, AWPPH may affect patients’ survival through factors other than tumor distant metastasis.

Correlation analysis indicates the involvement of AWPPH in tumor growth regulation, and *in vitro* cell proliferation analysis further confirmed this hypothesis. FZD7 as a critical player in Wnt pathway has pivotal functions in the regulation of cell proliferation in triple negative breast cancer [8]. In our study, we proved that AWPPH is likely an upstream positive regulator of FZD7 expression in the regulation of cell proliferation in triple-negative breast cancer. However, whether this regulatory role is direct or indirect is still unknown. It is worth to note that no significant changes in levels of FZD7 mRNA were observed after AWPPH overexpression. Therefore, AWPPH may affect FZD7 protein accumulation or degradation but not FZD7 gene transcription.

## Conclusion

In conclusion, AWPPH is likely an oncogenic lncRNA with up-regulated expression pattern in triple-negative breast cancer. AWPPH may participate in triple-negative breast cancer by promoting tumor growth but not tumor metastasis through the up-regulation of FZD7.

## Abbreviations

ER: estrogen receptor
FZD7: frizzled homolog 7
HER2: human epidermal growth factor receptor 2
LRP6: lipoprotein receptor-related protein 6
PR: progesterone receptor
